# Visuomotor Interactions and Perceptual Judgments in Virtual Reality Simulating Different Levels of Gravity

**DOI:** 10.3389/fbioe.2020.00076

**Published:** 2020-02-18

**Authors:** Barbara La Scaleia, Francesca Ceccarelli, Francesco Lacquaniti, Myrka Zago

**Affiliations:** ^1^Laboratory of Neuromotor Physiology, IRCCS Fondazione Santa Lucia, Rome, Italy; ^2^Department of Systems Medicine and Centre of Space Biomedicine, University of Rome Tor Vergata, Rome, Italy; ^3^Department of Civil Engineering and Computer Science Engineering, Centre of Space Biomedicine, University of Rome Tor Vergata, Rome, Italy

**Keywords:** internal models, visual perception, interceptive action, predictive processes, sensorimotor interactions

## Abstract

Virtual reality is used to manipulate sensorimotor interactions in a controlled manner. A critical issue is represented by the extent to which virtual scenarios must conform to physical realism to allow ecological human–machine interactions. Among the physical constraints, Earth gravity is one of the most pervasive and significant for sensorimotor coordination. However, it is still unclear whether visual perception is sensitive to the level of gravity acting on target motion displayed in virtual reality, given the poor visual discrimination of accelerations. To test gravity sensitivity, we asked participants to hit a virtual ball rolling down an incline and falling in air, and to report whether ball motion was perceived as natural or unnatural. We manipulated the gravity level independently for the motion on the incline and for the motion in air. The ball was always visible during rolling, whereas it was visible or occluded during falling before interception. The scene included several cues allowing metric calibration of visual space and motion. We found that the perception rate of natural motion was significantly higher and less variable when ball kinematics was congruent with Earth gravity during both rolling and falling. Moreover, the timing of target interception was accurate only in this condition. Neither naturalness perception nor interception timing depended significantly on whether the target was visible during free-fall. Even when occluded, free-fall under natural gravity was correctly extrapolated from the preceding, visible phase of rolling motion. Naturalness perception depended on motor performance, in addition to the gravity level. In sum, both motor and perceptual responses were guided by an internal model of Earth gravity effects. We suggest that, in order to enhance perceptual sensitivity to physical realism, virtual reality should involve visual backgrounds with metric cues and closed-loop sensorimotor interactions. This suggestion might be especially relevant for the design of rehabilitation protocols.

## Introduction

When controlled manipulations of sensorimotor interactions are required, virtual reality tools are now a preferred choice in both basic research and rehabilitation (e.g., Sveistrup, 2004; Sanchez-Vives and Slater, 2005; Bohil et al., 2011; Cano Porras et al., 2018). An important concern for the design of virtual scenarios is represented by the physical realism of biological and non-biological animations, such as their obedience to the laws of dynamics. A preliminary question, however, is whether healthy observers are sensitive to potential deviations from physical realism. For instance, the sense of presence, i.e., the sense of being in the virtual environment rather than the place in which the participant’s body is actually located, does not seem to depend on visual realism greatly (Sanchez-Vives and Slater, 2005).

On the other hand, one would expect that observers should be specifically sensitive to physical invariants, which humans are exposed to since birth. One such constraint is given by Earth gravity. Given its ubiquitous presence, one would expect that human perceptual systems are exquisitely tuned to its effects. For instance, humans should be able to detect minimal departures from veridical gravitational acceleration in visual scenes. However, the evidence that this is the case remains controversial (Zago and Lacquaniti, 2005; Ceccarelli et al., 2018; Jörges et al., 2018; Vicovaro et al., 2019). The issue is especially relevant in rehabilitation applications requiring visuomotor interactions of the patients with the virtual reality setup. The benefits of rendering realistic effects of gravity in the visual stimuli are not obvious, considering that the resulting motions might be so fast as to be challenging for the visual system and taking into account the poor discrimination of accelerations. Therefore, it becomes critical to know whether or not human observers are able to detect the congruence or incongruence of the stimuli with physical gravity. Cybersickness might become an issue in the affirmative case (Rebenitsch and Owen, 2016). In the following, we first review evidence in favor and against the hypothesis that humans take gravity effects into account in sensorimotor interactions.

The evidence for motor actions is uncontroversial. Thus, it is well established that humans take gravity effects into account to control reaching movements optimally (Gaveau et al., 2011, 2016), to guide locomotion on an inclined plane (Cano Porras et al., 2019), and to interact effectively with objects moving under Earth gravity (Zago et al., 2009; Lacquaniti et al., 2013). For instance, healthy participants easily intercept a target dropped vertically from above or rolling down an inclined plane, even with sparse visual information (e.g., Lee et al., 1983; Lacquaniti and Maioli, 1989a; Michaels et al., 2001; Zago et al., 2004; La Scaleia et al., 2014a). This indicates the ability to predict the future position of the target, compensating for ambiguous or impoverished visual information as well as for sensorimotor delays (100–200 ms to process visual information and to transmit the resulting motor commands to the muscles and limbs, McLeod, 1987; Bootsma and Van Wieringen, 1990; Day and Lyon, 2000; Marinovic et al., 2009; Vishton et al., 2010).

Since the visual system is poor at discriminating arbitrary accelerations (Calderone and Kaiser, 1989; Werkhoven et al., 1992), it has been argued that predictive mechanisms for accelerating targets are based on a prior model of motion, integrated with sensory information (e.g., Mrotek and Soechting, 2007; van Soest et al., 2010; Franklin and Wolpert, 2011; de Rugy et al., 2012; Tramper et al., 2013; Mischiati et al., 2015). In particular, it has been shown that an internal model of the effects of Earth gravity is used to predict the motion of an object normally accelerated by gravity (Lacquaniti and Maioli, 1989b; Lacquaniti et al., 1993; Tresilian, 1997; McIntyre et al., 2001; Zago et al., 2004, 2009; Indovina et al., 2005; Senot et al., 2005, 2012; La Scaleia et al., 2015; Jörges and López-Moliner, 2017; Smith et al., 2018).

Interceptions can still be accurate even when the target is virtual and it moves vertically or on a parabolic path under simulated Earth gravity in a visual scene with sufficient context cues about the environmental reference and metric scale, whereas the timing errors (TEs) increase considerably when the background scene lacks context cues (Miller et al., 2008) or the target moves under simulated levels of gravity departing from Earth gravity (Miller et al., 2008; Zago et al., 2011; Bosco et al., 2012; Russo et al., 2017; Jörges et al., 2018). Likewise, ocular tracking of a virtual target that moves on a parabolic path accelerated by Earth gravity is more accurate than tracking a target that moves at constant speed, hypo- or hyper-gravity (Delle Monache et al., 2019; Jörges et al., 2018).

While there is abundant evidence that models of the physical properties and forces are used in motor tasks, a more controversial question is whether they are used also in cognitive and perceptual tasks (Hubbard, 2018). Indeed, several studies have shown that people often do not have a good intuitive understanding of the physics of gravitational motion (Shanon, 1976; Champagne et al., 1980), and perceptual judgments tend to be flawed (Kozhevnikov and Hegarty, 2001). For instance, people are generally poor at detecting motion anomalies of artificial animations of a target descending along an incline (Bozzi, 1959, 1961; Vicario and Bressan, 1990; Hecht, 1993). Moreover, most people believe that heavier objects fall faster than lighter ones (Shanon, 1976; Champagne et al., 1980; Vicovaro, 2014; Vicovaro et al., 2019), despite motor timing in a catching task is invariant under wide changes of mass of the falling ball (Lacquaniti and Maioli, 1989b). Smith et al. (2018) showed that the extrapolation of ballistic pendulum motion is idiosyncratic and erroneous when people draw the trajectories, but consistent with accurate physical inferences under uncertainty when people must process pendulum trajectories to catch a ball or they release a pendulum to hit a target. Also, when observers were asked to judge which of two visually presented parabolic motions of a virtual target presented against a blank background had the higher simulated gravity, they generally showed high discrimination thresholds, suggesting that a prior of Earth gravity does not give rise to a discriminability of different gravity accelerations better than that for other arbitrary accelerations (Jörges et al., 2018).

The dissociation between high accuracy and precision in motor interception and low accuracy and precision in perception of gravitational motion seems consistent with the idea that priors may differ between perceptual and sensorimotor tasks (Chambers et al., 2019). However, the reason why perceptual and motor responses should rely on different strategies is still unclear. It has been proposed that visual information for action and visual information for perception involve different processes possibly mediated by distinct cerebral networks (dual-system hypothesis, e.g., Goodale and Milner, 1992; Jeannerod et al., 1995; Tresilian, 1995; Zago and Lacquaniti, 2005), but we still do not know when each process is called into play.

On the other hand, some studies showed that perception of static or dynamic stimuli may be affected by the assumption of gravity effects (Hubbard, 2018). Thus, perceptual processing of a target moving in different directions is affected by an internal model of the direction of Earth gravity (Miwa et al., 2019), as does the interpretation of biological motion (Troje and Chang, 2013; Maffei et al., 2015) and the processing of static configurations of human bodies (Barra et al., 2017). Also, when viewing a target that oscillates back-and-forth along a circular arc, observers perceive as uniform only kinematic profiles close to harmonic motion, consistent with the assumption of a pendulum accelerated by gravity (La Scaleia et al., 2014b). Moreover, stimuli moving downward at constant speed are perceived as faster than stimuli moving upward or rightward, consistent with the hypothesis that observers combine sensory measurements with a prior assumption of approximate gravity effects (Moscatelli et al., 2019). In addition, if the visual scene is rich of contextual cues providing an environmental reference and scale, the discrimination of time duration of accelerated targets is more precise for downward motion than for upward or horizontal motion (Moscatelli and Lacquaniti, 2011). In a recent study also involving a visual scene rich of contextual cues, participants watched the rolling motion of a sphere along a sloped path, and they adjusted the slope angle until the resulting motion looked natural for a given ball acceleration or adjusted the acceleration until the motion on a given slope looked natural (Ceccarelli et al., 2018). On average, participants were rather accurate at finding the match between slope angle and ball acceleration that was most congruent with physics. Therefore, implicit knowledge of gravity effects seems to play a role also in perceptual tasks, but it is still unknown whether and how it contributes to predictive processes affording perceptual extrapolations of object motion.

Here, we extend the findings of Ceccarelli et al. (2018) by investigating how knowledge of the effects of gravity is integrated with visual information in experiments requiring both the interception and the perceptual judgment of naturalness for targets moving under different levels of simulated gravity. Specifically, participants had two different tasks to accomplish during each trial. First, they tried to hit a virtual ball rolling down an inclined plane and then falling in air with different laws of motion. Immediately afterward, they were asked to report whether ball motion had been perceived as natural or unnatural.

We employed targets obeying two different kinematic laws in the two successive phases of descent, in order to probe the predictive nature of motion extrapolation (La Scaleia et al., 2015). Thus, the ball first rolled down in rectilinear motion along a 7°-incline accelerating at about 9% of the imposed gravity level, and then fell along a parabolic path at 100% of the same or different gravity level. Target kinematics during the falling phase cannot be extrapolated simply from visual information obtained during the rolling phase, but requires an internal model of free-fall as derived from prior knowledge.

We manipulated the ball acceleration for the motion on the inclined plane and for the motion in air independently, providing five experimental conditions. There were three internally consistent conditions (G_0_, G_1_, G_2_), in which the rolling phase on the plane was consistent with the falling phase in air, based on one of three different levels of gravity: Earth gravitational acceleration (g = 9.81 m/s^2^ for G_0_), half of this value (g/2 = 4.91 m/s^2^ for G_1_), or twice this value (2g = 19.62 m/s^2^ for G_2_). In two inconsistent conditions (G_3_, G_4_), instead, the motion on the plane was compatible with g, while the falling phase in air was at g/2 or 2g for G_3_ and G_4_, respectively. Therefore, only the condition G_0_ in which the gravity level was g during the entire ball motion—on the plane and in air—was compatible with a natural gravitational motion. In addition, there were two conditions of visibility of ball motion during the falling phase in air just before the interception, a visible and an occluded condition.

We manipulated the ball acceleration in order to explore if participants were able to modulate their behavior (interception and perceptual judgment) as a function of different gravity levels. We manipulated the visibility of the target during the falling phase to investigate if knowledge of gravity contributes to predictive processes in both motor and perceptual tasks, and if this knowledge can be updated based on visual information obtained during the rolling phase.

One can expect different results according to different, plausible hypotheses. If the internal model of Earth gravity accounts for a downward accelerated motion only qualitatively, we would expect that perceptual judgments should not differ significantly at different simulated gravity levels, given that in all experimental conditions, ball motion was accelerated in the downward direction. Moreover, according to this hypothesis, motor timing should be more accurate at lower terminal speeds of the target since these are generally easier to intercept for accelerating motion (Port et al., 1997), the conditions G_1_ and G_3_ being those that involved lower accelerations and lower terminal speeds than the other conditions.

If instead the internal model of gravity accounts for Earth gravitational kinematics quantitatively, we would expect that the condition G_0_ should be perceived as natural in a significantly higher number of cases than the other conditions, since G_0_ is the only condition involving accelerations compatible with Earth gravity effects throughout. Moreover, according to this hypothesis, motor timing should be accurate in G_0_, late in G_2_ and G_4_ (when target acceleration prior to interception is higher than the expected value of Earth gravity), and early in G_1_ and G_3_ (when target acceleration is lower than the expected value). Critically, if the internal model of Earth gravity affords predictive, anticipatory estimates of target motion, one would expect that both the interception and the perceptual judgment of naturalness should be little affected by the visibility of the target during the falling phase just prior to interception, because kinematics of free-fall under Earth gravity during visual occlusion can be extrapolated by the internal model starting from the preceding, visible phase of rolling motion along the incline (La Scaleia et al., 2015).

A third possibility is that the prior model of ball motion is updated by using online visual information of the rolling phase on the incline. An updated model might then be used to predict the subsequent falling phase in air. If so, perception rate of naturalness and interception timing should be similar in all three internally consistent conditions (G_0_, G_1_, G_2_), in which the rolling phase obeyed the same gravity constraint as the subsequent falling phase, and the performance should be significantly better than in the two inconsistent conditions (G_3_, G_4_), at least in the occluded session.

These experiments also allowed addressing the question whether the interception performance affects the subsequent perceptual judgment. If it does, one expects that perceptual responses are modulated by the motor performance, in addition to a potential modulation by the gravity level.

## Materials and Methods

### Participants

Sixteen subjects (seven females and nine males, 30.4 ± 6.4, years old, mean ± SD) were recruited to participate in the study. Sample size was determined *a priori* based on previous studies from our laboratory involving motor and perceptual protocols with an inclined plane (La Scaleia et al., 2014a, 2015; Ceccarelli et al., 2018), and on the effects observed in the participants (different from those of the present experiments) of a pilot study. Participant inclusion criteria were no past history of psychiatric or neurological diseases, normal or corrected-to-normal vision, right-handedness (as assessed by a short questionnaire based on the Edinburgh scale), height between 1.65 and 1.88 m, and correct responses in the preliminary tests carried out prior to the experiment (see section “Preliminary Tests”). The latter criteria had to be met to allow both an optimal view of the visual scene and the reachability of all targets in the workspace (see below). All participants were unaware of the experimental purpose and gave written informed consent to procedures approved by the Institutional Review Board of Santa Lucia Foundation, in conformity with the Declaration of Helsinki on the use of human subjects in research.

### Apparatus and Visual Stimuli

The participants sat on a height-adjustable chair in front of a mini-CAVE (Cave Automatic Virtual Environment) in a dark room. They wore shutter glasses and held a green cylindrical plastic object (size: 12 cm × 3 cm [height × diameter]; weight: 60 g), in the following denoted as the “hitter,” in the right hand (see Figure 1, inset) and a Wand Sensor (IS-900 system, InterSense Inc., Bedford, MA, United States) in the left hand used for button-press. The hitter had been realized with Ultimaker 2 + Extended 3D printer starting from a custom design with Autodesk. The mini-CAVE (VRMedia S.r.l., Pisa, Italy) consisted of four projection screens: a frontal screen 1.05 m wide and 1.05 high, two lateral screens 1.40 m wide and 1.05 m high, which were tilted by 15°23’ relative to the sagittal plane (to the left or right for the left and right screen, respectively), and a horizontal screen of trapezoidal shape (isosceles trapezoid) with 0.99 m height and bases length of 1.05 and 1.57 m (for the near and far side relative to the observer, respectively). All mini-CAVE walls were front-projection screens and the optic paths were halved by means of mirrors. Position and height of the chair were adjusted so that the eyes of each participant were located at a horizontal distance of about 0.95 m from the frontal screen and roughly centered on the frontal screen midpoint. The horizontal and vertical field of view (FOV) was about 180° and 160°, respectively. 3D visual scenario and stimuli were generated with XVR (eXtreme Virtual Reality, VRMedia S.r.l., Pisa, Italy, Tecchia et al., 2010), and were rendered in quasi-real time by an HP workstation Z210 with an ATI Firepro 3D V7900 graphics card (master PC). Two slaves HP workstations Z210 drove synchronously the 3D rendered graphical output to four LCD front projectors for screen display (3 NEC U300XG for the left, right, and frontal screen, ACER S5301WM DLP 3D-ready for the horizontal screen; 60-Hz stereo frame rate; 768 × 768 pixels resolution for the frontal screen, and 1024 × 768 pixels for the other screens).

**FIGURE 1:** Schematic of the experimental setup and visual scenario. The white lines and the gray area indicate the position of the mini-CAVE and the participant, respectively. The *x*,*y*,*z* reference system on the blue cuboid is shown for illustrative purpose only (it was not present in the virtual scene). The right inset shows the hitter held by the participant.

Head position and orientation were tracked online by means of the Vicon system (10 Bonita cameras). A bar (length × width × height 7 cm × 1.5 cm × 1.2 cm) equipped with four reflective spherical markers was placed on top of the bridge of the stereo shutter glasses. Position and orientation of the rigid body created from these markers were acquired at 100 Hz by the Vicon system to update the virtual scene based on head position and orientation. In separate tests, we measured an average update latency of three stereo frames.

Position and orientation of the hitter were also acquired at 100 Hz by the Vicon system. Three plastic pins protruded from the cylindrical body of the hitter, one of them (4.3 cm length, 0.7 cm diameter) was orthogonal to the cylinder axis and the others (1 and 3 cm length, 0.3 cm diameter) were parallel to it. An additional pin (1 cm length, 0.3 cm diameter) protruded from a winged frame fixed to the lower base of the cylinder. A reflective spherical marker was embedded on each pin-tip. 3D position and orientation of the hitter was reconstructed in real time from the position and orientation of the virtual rigid body connected by these markers, and from the known geometry of the hitter and its protruding parts. The coordinates of the objects monitored by the Vicon system were transformed in real-time into those of the virtual environment (XVR) by means of the calibration parameters obtained before the experiment. The calibration involved placing the Vicon test bar at several different locations in the experimental workspace and computing the translation vector and rotation matrix representing the transformation between the two coordinate systems. After the calibration, its accuracy was assessed with repeated acquisitions (*n* = 11) of an array of markers distributed in the workspace. On average, target registration error was 0.925 mm (± 1.052 SD), 0.470 mm (± 0.869 SD), and 0.412 mm (± 0.264 SD), for *x*, *y*, and *z* coordinates, respectively.

The scene background depicted part of a furnished laboratory (10.4 m wide, 13.2 m long, 3.10 m high in world scale), as a realistic version of the actual laboratory where the experiments were performed (Figure 1). The scene was projected at a 1:1 scale, with truthful width-depth rendering. Perspective geometry and textures were included in the scene to augment 3D effects. An inclined plane (2.5 m long, 0.15 m wide) supported by two tripods was placed with the lower edge 0.30 m to the left of the center line of the background wall; its longitudinal axis was parallel to the background wall. The incline was shown tilted by 7° relative to the horizontal. A textured, wooden ball (diameter, 8 cm), initially at rest over the plane, was released and rolled down the incline with different accelerations depending on the protocol, without slipping or bouncing. One static character imported from Autodesk 3ds Max 2010 was placed near the incline in the virtual laboratory to provide an additional metric reference for the virtual environment.

The hitter held by the subject during the experiment was truthfully displayed in the 3D virtual scene, except for the color of one marker on a reference pin-tip (reflexive gray color of the marker was displayed as orange in the virtual environment). Hitter display was necessary because hand interceptive movements occurred below the horizontal screen, remaining invisible to the participant. Spatial registration of the real hitter and its virtual image was obtained during the calibration phase.

### Ball Kinematics

Starting from rest, the ball rolled down the plane without slipping or bouncing. The simulated motion corresponded to that of a sphere with a homogenous mass distribution, accelerated by gravity and with negligible rolling resistance. Motion equation was:

(1) $$s\,\left(t,\theta \right)=\frac{1}{2}\cdot \frac{5}{7}\cdot a\cdot \left(\sin\theta \right)\cdot t^{2}$$

where *s* is the time-varying position of the center of mass of the ball along the plane axis, θ is the plane tilt relative to the horizontal (θ = 7°), and *a* is the gravity acceleration. During the experiment, *a* could take one of 3 different values g/2, g, or 2g (g = 9.81 m/s^2^).

Once the ball reached the lower end of the incline, it fell off the incline along a parabolic trajectory with acceleration *a* (we assumed negligible air drag and edge effects) and, once reached the floor, disappeared from the visual scene. The position of the ball center at the time the ball fell off the incline is denoted as the exit point. The height of the ball at the exit point was 1.05 m above the floor. The starting position of the ball on the incline and ball acceleration were randomized across trials. Notice that the inhomogeneous texture of the ball surface provided optical cues about the rotational component of the motion. The longitudinal axis of the inclined plane was parallel to the background wall, allowing the observer to see the entire trajectory of the ball. A hollow rectangular blue cuboid (1 m × 0.37 m × 0.085 m, length × height × width) contiguous to the lower edge of the incline was displayed on the visual scene. Its long axis, parallel to the background wall and to the floor, was placed in the frontal plane of motion of the ball center. The lower border of the cuboid was 32 cm below the center of the ball at the exit position from the incline, and the cuboid center was located 0.135 m below and 0.50 m to the right of ball exit point and it was at the same depth of ball exit point (see Figure 1). The cuboid had two open sides, the left side and the base, so that the ball could pass through the cuboid space without touching the walls. The first phase of parabolic motion of the ball was made either visible or occluded in separate sessions by making transparent or opaque the frontal side of the cuboid proximal to the participant.

The position of the observer in front of the scene was such that the midpoint between his/her eyes was 0.40 m above and 0.30 m to the right of the lower end of the incline, and 0.48 m in front of the incline longitudinal axis. The hitter held by the subject during the experiment was displayed in the 3D virtual scene as a cylindrical object very similar to the real one except for the color of the marker on the tip of the hitter (reflexive gray in the real, orange in the virtual one). This virtual object was rendered in real time and displayed in the same position as the hitter. The measured latency from the acquisition of 3D marker positions and video output ranged between 33 and 50 ms. The starting region of arm movements was rendered as a spherical volume in the 3D scene consisting of a white, partially transparent sphere (8 cm diameter) inscribed in a red cube 9 cm side, 0.60 m below, 0.60 m to the right, and 0.30 m in front of the ball exit point.

### Tasks

In each trial, a ball appeared at rest over the incline at a given initial position. To begin a trial, the participant placed the tip (orange marker) of the virtual hitter inside the starting region, and then pressed the Start button of the Wand Sensor. After a pseudorandom delay between 300 and 600 ms (in 100 ms steps), the ball rolled down the incline, fell off to the floor and disappeared from the visual scene. Participants were asked to hit the ball as soon as it emerged from the cuboid, neither the position nor the time of emergence being specified in advance. After the interception attempt and ball disappearance, participants were asked to give a two-alternative forced-choice judgment about the naturalness of the observed motion. To this end, they pressed one of two virtual buttons as a function of the chosen answer. The virtual buttons were created in the following way. After ball disappearance, as soon as participants moved the hitter at a frontal distance of 0.14 m from the ball exit point along the direction from the interception position to the starting position, two cubic white selection boxes (8 cm sides) were displayed in the visual scene. The two boxes were centered 0.20 m to the left and right of the center of the starting region for the hitter, 0.15 m above, and at 0.30 m frontal distance from the center (toward the incline). Frontal faces of the left and right box were labeled with capital letter “N” and “I,” respectively. Participants were required to enter the hitter inside the “N” box if the observed motion appeared as a natural motion (N is the initial letter of the Italian word “naturale”), or inside the “I” box if the observed motion appeared as an unnatural motion (“I” is the initial letter of the Italian word “innaturale”). Subjects were instructed to provide a judgment about the entire ball trajectory, taking into account both the rolling phase and the parabolic phase of ball motion. Once the hitter was entered within one box, the box color changed from white to orange.

#### Preliminary Tests

Before the beginning of the first experimental session, adequate visual acuity in the 3D virtual environment and ability to reach specified targets were tested. Correct responses to the preliminary tests were required to include a subject in the experiment. Using these criteria, no subject was excluded from the study. Neither the inclined plane nor the blue cuboid displayed in the subsequent experiment was shown during the preliminary tests. Instead, different types of objects were shown.

##### Stereopsis and color vision

To assess whether participants could see the 3D objects projected on the screens, subjects were asked to wear shutter glasses and to watch a scene in the mini-CAVE in which three red and two green spheres (radius 7.5 mm) were displayed in front of them at 0.48 m distance from the midpoint between the eyes. The spheres were at 0.10 m horizontal and vertical distance between each other. Subjects were asked to count the number and indicate the color of the spheres displayed on the frontal screen.

##### Reachability of the workspace

Here, a cuboid grid of 20 yellow spheres (5 mm radius) was projected on the screens to the right of the position of the inclined plane in the actual experiment. The distance between the proximal spheres in the grid was 0.1 m horizontal, 0.04 m vertical, and 0.045 m in depth, along the axis *x* (see reference system in Figure 1). Size, position, and orientation of the cuboid grid were the same as those of the blue cuboid of the experiments, except that the vertical quote of the cuboid grid was centered on the starting spherical volume of the hitter, so as to test the reachability of the whole space covered by potential hitter movements in the subsequent experiment (starting region, interception space, judgment-task region). Participants were asked to hold the hitter and place its tip in the starting region as in the subsequent experiment. The test of reachability started once one of the spheres in the grid turned red and subjects were required to reach the red sphere with the hitter. After the reaching movement, the red sphere turned yellow again and another sphere in the grid turned red. Each of the 20 spheres was tested once for reachability. This task lasted about 1 min.

#### Familiarization Tasks

Three different tasks were carried out in the following sequence.

##### Ball hitting

Subjects were instructed to hit a static ball (same appearance and size as in the subsequent experiment) with the tip of the hitter. When the ball was hit, it turned red, a beep was emitted, and then the ball appeared in a different position. The ball could be placed at one of eight different positions, quasi-randomly selected, spaced so as to cover the interception region of the experiment. The spheres were positioned according to a grid (not showed in the scene), at a distance of 0.48 m from the midpoint between the eyes, along *z* axis, at a distance of 0.2 m from each other, along the axis *x*, centered on the starting position of the hand. The ball was placed once in each position.

##### Depth of ball trajectory

In the next task, a ball at the exit point of the inclined plane of the subsequent experiment and three different planes appeared in the virtual scene. One green plane (about 1.30 m × 0.08 m, height × wide) was perpendicular to the inclined plane. The other two planes (one red and the other blue, 1.23 m × 1 m, length × height) were parallel to the frontal plane, located at a distance of 0.08 m from each other, at a distance of 0.52 and 0.44 m, respectively, along *z* axis, from the midpoint between the eyes and centered on the plane of motion of the ball center during the subsequent experiment. Using the hitter, participants were instructed to explore visually and manually the space on the right side of the inclined plane. The green virtual object, depicting the hitter, turned gray when it entered the space between the two planes parallel to the frontal plane. This color change was used to give an indication of the depth of the virtual environment.

##### Interception and two-choice judgment task

In the last task, the ball was initially attached at the ceiling at about 0.38 m above, 0.21 m to the right and at a distance of 0.48 m along the *z* axis relative to the midpoint between the eyes of participant. When the subject pressed a button of the Wand Sensor, the ball fell vertically under gravity. The task was to hit the ball and then judge whether the motion appeared natural or unnatural, even though ball acceleration was always equal to g. Hitting and judgment were performed with a similar procedure as in the actual experiment (see above). After five such trials, the experiment began.

Overall, the familiarization phase lasted about 5 min and preceded each experimental session.

### Protocol

Participants were tested in a counterbalanced order in two sessions, occluded and visible, 15 days apart. In each session, there were 15 test conditions: three different starting positions of the ball on the incline, corresponding to three traveled distances (TD), and five different gravity conditions (G). TD corresponds to the distance between the starting and the exit position on the incline. The conditions are detailed in Table 1. The starting position of the ball and traveled distance on the inclined plane were calculated from the law of motion of a ball rolling down the plane without slipping or friction according to Eq. 1. We used the following combinations of gravity level for the rolling phase and gravity level for the falling phase in air (see Table 1). G_0_: g ÷ g. G_1_: g/2 ÷ g/2. G_2_: 2g ÷ 2g. G_3_: g ÷ g/2. G_4_: g ÷ 2g.

**TABLE 1:** Ball motion parameters (inclined plane and air).

**Gravity Condition**	**Inclined plane**				**Air**		
	**Gravity acceleration**	**Traveled distance**	**Motion duration**	**Speed**	**Gravity acceleration**	**Motion duration**	**Speed**
**#**	**[m/s^2^]**	**[m]**	**[s]**	**[m/s]**	**[m/s^2^]**	**[s]**	**[m/s]**
G_0_	g	0.546	1.13	0.96	g	0.244	2.69
G_0_	g	1.093	1.60	1.36	g	0.240	2.85
G_0_	g	2.186	2.26	1.93	g	0.233	3.16
G_1_	g/2	0.546	1.60	0.68	g/2	0.345	1.90
G_1_	g/2	1.093	2.26	0.96	g/2	0.339	2.02
G_1_	g/2	2.186	3.20	1.36	g/2	0.329	2.24
G_2_	2g	0.546	0.80	1.36	2g	0.173	3.80
G_2_	2g	1.093	1.13	1.93	2g	0.170	4.03
G_2_	2g	2.186	1.60	2.73	2g	0.165	4.47
G_3_	g	0.546	1.13	0.96	g/2	0.339	2.02
G_3_	g	1.093	1.60	1.36	g/2	0.329	2.24
G_3_	g	2.186	2.26	1.93	g/2	0.317	2.62
G_4_	g	0.546	1.13	0.96	2g	0.175	3.68
G_4_	g	1.093	1.60	1.36	2g	0.173	3.79
G_4_	g	2.186	2.26	1.93	2g	0.170	4.03

*The motion duration and the traveled distance on the inclined plane are from the starting position until the end of the inclined plane. Speed is referred at the end of the inclined plane. The motion duration in the air is until the lower border of the box. Speed is at the exit of the box. For each gravity condition (G_0_–G_4_) is indicated the gravity acceleration acting on ball during the rolling phase on the inclined plane and the falling phase in the air.*

Each experimental session involved two identical blocks of 105 trials. In each block, there were 90 test trials and 15 catch trials (CTs), one for each test conditions, pseudo-randomly interleaved between the test trials, with unexpectedly altered visibility condition. For test trials, TD was assigned to one of three values, and G was assigned to one of five values. Each CT had the same TD and G as in the previous test trial, but a different visual condition (occluded if the test was visible or viceversa). In each block, targets were presented in consecutive sequences in which each test condition (3 TD × 5 G) was presented in random order, different from one sequence to the next. There were six such sequences (repetitions). In the first sequence of the block (first repetition) no test condition has a corresponding CT. In each of the other five sequences of block, there were three different test conditions with corresponding CTs (for a total of 15 CTs = 3 CTs × 5 sequences). Thus, each block had 105 trials [3 TD × 5 G × 1 R + (3 TD × 5 G + 3 CT) × 5 R], resulting in a total of 210 trials for each experimental session.

Figure 2 shows the last segment of the paths of the ball, while Figure 3 shows the time course of the center of mass. Notice that the internally consistent conditions (in blue) involved the same spatial trajectories of the ball but with a different time course.

**FIGURE 2:** Spatial trajectories of the ball for all experimental conditions. The envelope of the path followed by the ball in the frontal plane is denoted by parallel lines. Black lines indicate the last segment of the rolling motion on the inclined plane. Blue, red, and green lines indicate the trajectories in air for the internally consistent conditions (G_0_, G_1_, G_2_), the inconsistent condition G_3_, and the inconsistent condition G_4_, respectively. The black box represents the frontal side of the cuboid. Each panel corresponds to a different traveled distance (TD) on the incline.

**FIGURE 3:** Time course of ball motion for all experimental conditions. Time-varying trajectories of the center of ball mass in the horizontal and vertical direction are plotted in the top and bottom rows, respectively, from the starting position on the incline to the arrival time of the ball on the virtual floor. Black lines indicate the motion on the incline. Blue, red, and green lines indicate the trajectories in air for the internally consistent conditions (G_0_ as continuous line, G_1_ asterisk-dashed, G_2_ dashed), the inconsistent condition G_3_, and the inconsistent condition G_4_, respectively. Each column corresponds to a different traveled distance (TD) on the incline.

A motivational score (10 points for each hit ball) was provided to the participants after each set of 15 trials, but subjects were unaware of the criterion used to score their performance.

Participants were allowed to pause any time they wished during an experimental session, which lasted about 32 min.

### Data Analysis

We excluded a few trials (∼4% of all trials) from the analysis due to the presence of artifacts or lack of subject’s attention (as marked in the experiment notebook). The 3D coordinates (*x*, *y*, *z*) of the tip of the hitter recorded by Vicon were numerically low-pass filtered (bidirectional, 20-Hz cutoff, second-order Butterworth filter). These data, as well as the position of the ball center, were interpolated at 1 kHz using a spline cubic interpolation.

#### Perceptual Task

##### Naturalness judgments

Perception rate of natural motion (PR) was computed as the proportion of trials in which participants judged the ball motion as natural relative to the total number of trials for each experimental condition of each participant. Thus perceptual responses were cumulated over all repetitions of each condition.

#### Motor Task

For each trial, we computed the following parameters.

##### Endpoint analysis

The minimum distance point (IP) was defined as the position in which the tip of the hitter (in the following, simply the hitter) first arrived at the minimum distance from the ball surface during ball motion. We also computed the time sample in which the trajectory of the hitter crossed, for the first time, the frontal plane tangent to the ball surface facing the hitter (i.e., when the ball could be intercepted for the first time). The TE was defined as the difference between the time sample when the hitter crossed the frontal plane tangent to the ball surface and the time sample when the hitter reached IP. Accordingly, a positive (negative) value of TE corresponded to a response later (earlier) than that theoretically expected if the hitter arrived at a minimum distance from the ball when crossing the frontal plane tangent to the ball surface facing the hitter. The schematic of Figure 4 shows the top view of hypothetical hand trajectories, when the interception movement of the hitter is timed early relative to ball arrival (Figure 4A), when it is timed accurately (Figure 4B), or when it is timed late (Figure 4C).

**FIGURE 4:** Top view of the relative position of the ball and hand in three hypothetical cases. Each panel is a snapshot representing the relative position of the ball and hitter in the horizontal plane at a given time. The gray region delimits the proximal and distal frontal planes tangent to ball surface. The blue lines depict the paths that led the hitter at the position depicted in the panel. The black cross denotes the position IP in which the hitter first arrived at the minimum distance from the ball surface during ball motion. The purple circle denotes the position of the hitter when it first crossed the proximal frontal plane tangent to the ball surface. **(A)** The hitter arrives early relative to the ball, and the timing error (TE) is negative. **(B)** The hitter arrives on time (TE = 0). **(C)** The hitter arrives late (TE > 0).

##### Comparison with natural gravitational free-fall in air

We computed the virtual ball parabolic trajectory in air under natural gravity (gravitational ball trajectory), independently of the previous ball acceleration during the rolling motion on the incline. We defined the gravitational timing error (GTE) as the difference between the time sample when the hitter crossed the frontal plane tangent to the ball surface and the time sample when the hitter reached the minimum instantaneous distance from the ball surface, assuming a free-fall under natural gravity (instead of the actual kinematics in the current trial). GIP was defined as the corresponding virtual minimum distance point. Accordingly, if participants predicted a free-fall of the ball in air under natural gravity, GTE should be zero and GIP should be independent of the previous ball acceleration during the rolling phase.

##### Hand kinematics

We considered the time-varying position of the hitter, which was time-differentiated to compute the tangential speed as *v*_T_ = $\sqrt{\left({\dot{x}}^{2}+{\dot{y}}^{2}+{\dot{z}}^{2}\right)}$. We computed the maximum tangential speed of the hitter during the entire hand movement and the interval between the time sample in which the hitter arrived in IP and the time sample of maximum speed. Onset time of hand movements was computed according to the following algorithm (La Scaleia et al., 2015). First, we normalized tangential speed to the maximum value v = v_T_/v_*max*_. Then, going back from the time sample at which v = 1, we defined the first sample for which v ≤ 0.08 as the onset time. We defined movement duration (MD) as the interval between the onset time and the time of maximum speed.

### Statistical Analysis

The main statistical analyses excluded the CTs, so we considered 12 repetitions (six repetitions per block) for each experimental condition. CTs were included in a separate analysis, as a control for the effect of visibility condition. Results are reported as mean and 95% confidence intervals (CIs) for data symmetrically distributed. Perception rate of natural motion (PR, binary responses) is reported as quartiles (median and interquartile range, IQR = q3 – q1 where q1 and q3 are the 25th and 75th percentiles). Perception rates higher than q3 + 1.5(q3 – q1) or smaller than q1 – 1.5 (q3 – q1) were considered as outliers.

For perception rate of natural motion, the statistical differences between conditions were assessed using a generalized linear mixed model (GLMM, see Moscatelli et al., 2012) with logit link function. GLMM separates the overall variability into a fixed component and a random component, and assumes that the response variable has a binomial distribution. The fixed component estimates the experimental effect, while the random component estimates the heterogeneity between participants. We considered the following model:

logit[P(Y=ij1)]=δ+0u+j0(δ+1u)j1G+(δ+2u)j2TD+(δ+3u)j2V+δO4+δTD5×G

In this model, the logit transformation of the probability that participant j judged natural the ball motion in trial i is equal to a linear combination of fixed and random effect predictors. Specifically, **G** is the categorical variable for the Gravity Condition (G = G_0_, G_1_, G_2_, G_3_, G_4_), **TD** is the categorical variable for the traveled distance on the incline (TD = TD0, TD1, and TD2 for starting position 0.546, 1.093, and 2.186 m, respectively), **V** is the dummy variable for the visual condition (V = 0 or 1 for the occluded or the visible condition, respectively), and **O** is the dummy variable for the session order (O = 0 or 1 if the first experimental session was visible or occluded, respectively). **TD** × **G** is the interaction between the traveled distance on the incline and gravity condition. δ_k_ are the fixed effects coefficients and u_jk_ are the random effects coefficients.

To analyze the correlation between perceptual and motor responses, we included in the model (Eq. 2) the absolute value of the TE [continuous variable, δ_6_ abs(**TE**)] as predictor. The abs(TE) is related to the relative success of the interceptive action: the lower the value of abs(TE), the higher the relative success.

The significance of fixed effect parameters was assessed by means of Wald statistics. We selected each GLMM model from a pool of nested models based on the Akaike information criterion.

The TE and all other kinematic parameters were modeled using a linear mixed model (LMM), which is a special case of the GLMM assuming an identity link function. In LMM, the response variable is assumed to have a conditional Gaussian distribution. The response variable is modeled as a linear combination of the fixed-effect and random-effect parameters.

In the LMM model, we included the repetitions (R, continuous variable) as a predictor [(δ_7_ + u_j__7_) **R**].

All analyses were performed in Matlab (Mathworks, Natick, MA, United States) and R environment (R Development Core Team, 2011; R Foundation for Statistical Computing, Vienna, Austria).

## Results

### Perception Rate of Natural Motion

In each trial, the ball rolled down an incline and then fell off in air with different kinematics, depending on the test condition (Figures 1–3 and Table 1). After trying to intercept the ball exiting from the cuboid, participants provided a two-alternative forced-choice judgment about the perceived naturalness of the previous motion of the ball. We found that perception rate of natural motion (PR) was significantly higher and less variable (across participants, starting positions of the ball, and visual conditions, visible or occluded) in G_0_, the only condition in which ball kinematics was congruent with Earth gravity during both the rolling phase and the free-falling phase, than in all other conditions (Figure 5). Thus, PR for G_0_ was 83.3% (IQR = 26.14%, three traveled distances × two visual conditions × 16 subjects, *n* = 96), while it was 66.7% (IQR = 74.24%), 26.8% (IQR = 49.2%), 58.3% (IQR = 58.3), and 41.7% (IQR = 41.7%) for G_1_–G_4_, respectively.

**FIGURE 5:** Perception rates of natural motion plotted separately for each gravity condition (three traveled distances × two visual conditions × 16 subjects, *n* = 96). The bottom and top of the box-and-whisker plots boxes correspond to the lower and upper quartile, respectively. The notch displays the 95% confidence interval of the median. The whiskers extend to the lowest and highest data points, without considering the outlier (cross).

To take into account the variability across participants, we used the GLMM with gravity condition G_0_, traveled distance on the incline TD1, visibility: Occluded, and session order: Occluded in the first block, as the baseline conditions in Eq. 2. This analysis showed that PR depended significantly on gravity conditions and on the interaction between gravity conditions and traveled distance (Figure 6 and Table 2). In particular, PR was significantly higher for G_0_ than for all other conditions (all coefficients for G_1_–G4 were negative, implying that their values were lower than the PR of the baseline, see Eq. 2). These differences were significant for all gravity conditions G_1_–G_4_ (all *P* < 0.024). Therefore, neither the internal consistency of the gravity level between the rolling phase and the falling phase in air (G_1_–G_2_) nor the congruence of the rolling phase with natural gravity g (G_3_–G_4_) was sufficient to judge the movement as natural in a systematic way. Furthermore, PR did not depend significantly on visibility (*P* = 0.261), but it was significantly lower when the first session was occluded than when it was visible (*P* < 0.0001).

**FIGURE 6:** Perception rates of natural motion for each gravity condition, visual condition, and traveled distance on the incline (*n* = 16 subjects). Different gray levels denote different traveled distances: 0.546, 1.093, and 2.186 m, dark to light. Other conventions as in Figure 5.

**TABLE 2:** Natural perception rate.

	***Coeff***	***P*-value**
Intercept	1.26	4.13E−06***
TD0	0.30	0.188
TD2	–0.12	0.594
G_1_	–0.99	0.024*
G_2_	–2.48	2.28E−10***
G_3_	–1.27	3.51E−05***
G_4_	–1.76	4.48E−07***
Visibility (V)	–0.18	0.261
Session order (O)	0.89	5.23E−05***
TD0 × G_1_	–0.05	0.849
TD2 × G_1_	–0.46	0.087
TD0 × G_2_	–0.48	0.077
TD2 × G_2_	0.46	0.087
TD0 × G_3_	0.43	0.103
TD2 × G_3_	–2.00	2.84E−13***
TD0 × G_4_	–0.97	0.0002***
TD2 × G_4_	0.48	0.052

All coefficients of the GLMM for the fixed factors in the model used to fit the natural perception rate reached by participants and the relative *P-value* values are shown (gravity condition G_0_, traveled distance TD1, visibility: occluded, and session order: occluded in the first block are the baseline). ***P < 0.001.

To analyze the correlation between perceptual and motor responses, we included the absolute value of the TE of interception (TE, continuous variable, see next section) as a predictor in the model. The GLMM analysis showed that PR decreased significantly with increasing absolute value of TE (*P* = 0.012, Table 3). Furthermore, this analysis confirmed that PR was higher when ball kinematics was congruent with Earth gravity (G_0_) throughout descent than when it was not (all coefficients for G_1_–G4 were negative, and all *P* < 0.032).

**TABLE 3:** Correlation between perceptual and motor responses.

	***Coeff***	***P*-value**
Intercept	1.37	8.18E−07***
abs(TE)	–1.22	0.012*
TD0	0.30	0.188
TD2	–0.13	0.569
G_1_	–0.95	0.032*
G_2_	–2.48	1.61E−10***
G_3_	–1.25	4.50E−05***
G_4_	–1.74	6.05E−07***
Visibility (V)	–0.19	0.240
Session order (O)	0.89	6.22E−05***
TD0 × G_1_	–0.05	0.861
TD1 × G_1_	–0.45	0.098
TD0 × G_2_	–0.47	0.083
TD2 × G_2_	0.45	0.094
TD0 × G_3_	0.44	0.095
TD2 × G_3_	–2.00	3.65E−13***
TD0 × G_4_	–0.95	0.0003***
TD2 × G_4_	0.46	0.060

All coefficients of the GLMM for the fixed factors in the model used to fit the natural perception rate reached by participants and the relative *P-value* values are shown (gravity condition G_0_, traveled distance TD1, visibility: occluded, and session order: occluded in the first block are the baseline). ***P < 0.001.

In sum, perceptual judgments of naturalness depended in part on the gravity conditions and in part on the relative success of the interceptive action.

### Timing Error of Interception

The TE varied considerably as a function of the different gravity conditions (Figures 7, 8A). On average, TE was not significantly different from zero for G_0_ (TE = -0.014 ± 0.016 s, mean ± CI, *n* = 96, three traveled distances × two visual conditions × 16 subjects). Instead, mean TE was significantly negative, implying early responses, when the acceleration during fall in air was equal to g/2 (TE = -0.089 ± 0.020 s and TE = -0.085 ± 0.016 s, mean ± CI, *n* = 96, for G_1_ and G_3_, respectively). By contrast, mean TE was significantly positive, implying late responses, when the acceleration during fall in air was equal to 2 *g* (TE = 0.047 ± 0.014 s and TE = 0.059 ± 0.018 s, mean ± CI, *n* = 96, for G_2_ and G_4_, respectively).

**FIGURE 7:** Timing errors for each gravity condition and traveled distance on the incline (mean ± 95% confidence interval, two visual conditions × sixteen subjects, *n* = 32). Different gray levels denote different traveled distances as in Figure 6.

**FIGURE 8:** Timing errors and hand movement characteristics. **(A)** Timing errors (mean ± 95% confidence interval, three traveled distances × two visual conditions × 16 subjects, *n* = 96). **(B)** Intervals (mean ± 95% confidence interval, three traveled distances × two visual conditions × 16 subjects, *n* = 96) between the time at which the hitter arrived in IP and the time of maximum hitter speed. **(C)** Top view of hitter trajectories for all repetitions (*n* = 12) of a representative participant (#13) for each gravity condition and traveled distance (red 0.564 m, green 1.093 m, and blue 2.186 m) in the occluded session. The trajectories are plotted from the starting position to IP. Gray area represents the envelope of ball trajectory. **(D)** Speed profiles of hitter movements of the same subject of **C**. The 95% confidence interval over all repetitions and traveled distances in the occluded session are plotted for each gravity condition. Traces are aligned on the hitter arrival time in IP (vertical line).

A visual impression of these results with TE is provided by Figure 8C, showing the top view of hand trajectories for all repetitions of a representative participant for each gravity condition and traveled distance of the ball on the incline in the occluded session. The trajectories are plotted from the starting position to IP. A positive (negative) value of *z*-coordinate of IP indicates late (early) responses, whereas *z*-coordinates close to 0 (the *z*-coordinate of the frontal plane tangent to the ball surface facing the hitter) indicate correctly timed responses (see also Figure 4). It can be seen that most hand movements aimed at targets accelerating at g/2 during fall in air (G_1_ and G_3_) were early, those aimed at targets accelerating at 2 *g* (G_2_ and G_4_) were late, and those aimed at targets accelerating at g (G_0_) were mostly on time.

Linear mixed model (five gravity conditions, three traveled distances, twelve repetitions, two visual conditions, and two session orders) confirmed the results. TE depended significantly on gravity condition (all *P* < 10^–19^, Table 4). TE was not significantly different from zero (*P* = 0.150) for G_0_, whereas the coefficients for G_1_ and G_3_ (G_2_ and G_4_) were negative (positive), indicating early (late) responses relative to the responses in G_0_. TE did not depend significantly on visibility, repetitions, or session order (all *P* > 0.080). Similar results were obtained by including also CTs. In order to evaluate their potential effect, we compared the TE of consecutive trials with the same traveled distance and gravity condition but different visual condition. In particular, for each CT, we evaluated the difference between the TE of an occluded trial and the TE of the corresponding visible trial, independently of presentation order. Table 5 shows that in the occluded session the visibility did not change the TE (*P* = 0.989).

**TABLE 4:** Timing error.

	***Coeff***	***P*-value**
Intercept	–31.38	0.150
TD0	15.34	0.016*
TD2	–11.60	0.065
G_1_	–72.34	1.42E−19***
G_2_	74.40	4.45E−26***
G_3_	–68.04	1.78E−31***
G_4_	76.97	2.88E−39***
Visibility (V)	28.50	0.080
Session order (O)	26.18	0.162
Repetition	–1.61	0.257
TD0 × G_1_	–9.94	0.183
TD2 × G_1_	3.07	0.684
TD0 × G_2_	–1.18	0.875
TD2 × G_2_	–37.12	1.29E−06***
TD0 × G_3_	–14.25	0.056
TD2 × G_3_	8.32	0.271
TD0 × G_4_	8.43	0.259
TD2 × G_4_	–19.28	0.011*

All coefficients in milliseconds of the LMM for the fixed factors in the model used to fit the timing error and the relative *P-value* values are shown (gravity condition G_0_, traveled distance TD1, visibility: occluded, and session order: occluded in the first block are the baseline). *P < 0.05, ***P < 0.001.

**TABLE 5:** Effect of “catch trials” on timing error.

	***Coeff***	***P*-value**
Intercept	0.16	0.989
TD0	–7.50	0.631
TD2	0.20	0.990
G_1_	0.97	0.956
G_2_	–10.76	0.466
G_3_	6.54	0.668
G_4_	–3.27	0.838
Visibility (V)	16.22	0.054
Session order (O)	11.44	0.102
TD0 × G_1_	0.42	0.984
TD2 × G_1_	–2.02	0.923
TD0 × G_2_	26.06	0.206
TD2 × G_2_	–5.52	0.797
TD0 × G_3_	–4.97	0.810
TD2 × G_3_	5.72	0.787
TD0 × G_4_	–12.46	0.545
TD2 × G_4_	6.41	0.759

*All coefficients in milliseconds of the LMM for the fixed factors in the model used to fit the timing error and the relative *P-value* values are shown (gravity condition G_0_, traveled distance TD1, visibility: occluded, and session order: occluded in the first block are the baseline).*

### Hand Kinematics

#### Spatial Scatter of Endpoints

Figure 9 plots for all trials the position of the hitter when it crossed, for the first time, the proximal plane tangent to the ball surface (i.e., when the ball could be intercepted for the first time). From Figure 2, we recall that the three internally consistent conditions (g-g, g/2-g/2, 2g-2g) involved the same spatial trajectories of the ball. Figure 9 shows that the corresponding endpoints of hand movements tended to be closely scattered along the trajectory of the ball for both visual conditions, indicating that subjects were generally able to extrapolate the target trajectory even when this was occluded from view. Remarkably, the endpoints of the movements in the two inconsistent conditions (g-g/2, g-2g) tended to fall in roughly the same region as those of the consistent conditions, therefore deviating conspicuously from the actual path of the ball.

**FIGURE 9:** Spatial distributions of endpoint positions. Each panel plots the *x*–*y* positions (*n* = 192) of the hitter when it crossed, for the first time, the proximal, frontal plane tangent to the ball surface for all trials of all participants in the indicated gravity condition. Curved parallel lines represent the envelope of the path followed by the ball in the frontal plane.

#### Interval Between the Instant in Which Hitter Arrived in the Minimum Distance Point and the Maximum Speed Time

The mean maximum speed was equal to 1.733 ± 0.097, 1.622 ± 0.090, 1.814 ± 0.105, 1.700 ± 0.094, and 1.756 ± 0.110 m/s (mean ± CI, *n* = 96, three traveled distances × two visual conditions × sixteen subjects) for G_0_–G_4_, respectively. The maximum speed was significantly greater in G_2_ (G_1_ and G_3_) (smaller) than in G0 (*P* < 0.02).

The mean time interval between the instant in which the hitter arrived in IP and the instant of maximum speed (IT) depended significantly on gravity condition: this interval was equal to 0.057 ± 0.022, 0.137 ± 0.027, -0.008 ± 0.020, 0.127 ± 0.022, and -0.015 ± 0.024 s (mean ± CI, *n* = 96) for G_0_–G_4_, respectively. Figure 8B plots this time interval for G_0_–G_4_. Table 6 shows the results of LMM (five gravity conditions, three traveled distances, twelve repetitions, two visual conditions, and two session order). The hitter arrived in IP after the maximum speed time in G_0_ (P = 0.001). The interval time depended significantly on gravity condition (*P* < 10^–21^), in particular in G_1_ and G_3_ (G_2_ and G_4_) the interval was greater (smaller) than in G_0_. Figure 8D shows the speed profiles (95% CI over all repetitions and traveled distances) of the hand movements of a representative subject (same as in Figure 8C) for each gravity condition in the occluded session, aligned with the hand arrival time in IP. The interval time did not depend significantly on visibility (*P* = 0.113).

**TABLE 6:** Interval between the instant in which hitter arrived in intersection point and the maximum speed time.

	***Coeff***	***P*-value**
Intercept	90.68	0.001**
TD0	–5.64	0.472
TD2	4.34	0.561
G_1_	75.78	1.120E−21***
G_2_	–81.77	7.35E−23***
G_3_	63.83	2.23E−22***
G_4_	–74.07	1.42E−29***
Visibility (V)	–28.74	0.113
Session order (O)	–64.87	0.004**
Repetition	1.87	0.110
TD0 × G_1_	22.64	0.008**
TD2 × G_1_	–10.52	0.220
TD0 × G_2_	2.52	0.767
TD2 × G_2_	47.57	5.02E−08***
TD0 × G_3_	20.82	0.014*
TD2 × G_3_	–3.71	0.666
TD0 × G_4_	–10.58	0.214
TD2 × G_4_	16.70	0.052

All coefficients, in milliseconds, of the LMM for the fixed factors in the model used to fit the gravitational timing error and the relative *P-value* values are shown (gravity condition G_0_, traveled distance TD1, visibility: occluded, and session order: occluded in the first block are the baseline). *P < 0.05, **P < 0.01, ***P < 0.001.

#### Movement Duration

The MD varied as a function of gravity conditions. On average, hand movements aimed at balls rolling down the incline with a higher acceleration lasted less than those aimed at balls with lower accelerations. On average, MD was 0.313 ± 0.014, 0.348 ± 0.017, 0.287 ± 0.012, 0.313 ± 0.015, 0.317 ± 0.016 s (mean ± CI, *n* = 96, three traveled distances × two visual conditions × 16 subjects) for G_0_–G_4_ respectively. LMM (five gravity conditions, three traveled distances, twelve repetitions, two visual conditions, and two session order) showed that MD depended significantly on gravity condition during the rolling phase on the incline (Table 7). In fact, the coefficients for G_3_ and G_4_ were not significantly different from zero (*P* > 0.686), indicating that, irrespectively of the gravity level during the falling phase in air, the hand movement had the same duration for gravity conditions G_0_, G_3_, and G_4_. By contrast, the hand movement lasted less (more) in G_2_ (G_1_) than that in G_0_. MD did not depend significantly on visibility (*P* = 0.235).

**TABLE 7:** Hand motion duration.

	***Coeff***	***P*-value**
Intercept	305.43	2.69E−64***
TD0	16.97	0.047*
TD2	–10.70	0.198
G_1_	35.44	1.75E−06***
G_2_	–25.82	0.0005***
G_3_	3.19	0.686
G_4_	2.52	0.726
Visibility (V)	–12.10	0.235
Session order (O)	–1.09	0.952
Repetition	1.62	0.126
TD0 × G_1_	–1.23	0.891
TD2 × G_1_	1.40	0.877
TD0 × G_2_	–10.05	0.264
TD2 × G_2_	7.80	0.398
TD0 × G_3_	–3.03	0.736
TD2 × G_3_	–5.29	0.561
TD0 × G_4_	3.71	0.681
TD2 × G_4_	0.01	0.999

All coefficients, in milliseconds, of the LMM for the fixed factors in the model used to fit the gravitational timing error and the relative *P-value* values are shown (gravity condition G_0_, traveled distance TD1, visibility: occluded, and session order: occluded in the first block are the baseline). *P < 0.05, ***P < 0.001.

This was confirmed also by the analysis of CTs. For both the MD and IT, we evaluated the differences between the value in the occluded trial and the corresponding one in the visible trial, independently of presentation order. In both visible and occluded sessions, visibility did not affect significantly either IT (*P* = 0.823, Table 8) or MD (*P* = 0.088, Table 9).

**TABLE 8:** Effect of “catch trials” on interval between the instant in which hitter arrived in intersection point and the maximum speed time.

	***Coeff***	***P*-value**
Intercept	3.05	0.823
TD0	3.86	0.827
TD2	–2.74	0.877
G_1_	–1.08	0.955
G_2_	11.91	0.490
G_3_	1.56	0.934
G_4_	3.88	0.824
Visibility (V)	–6.82	0.522
Session order (O)	–15.66	0.049*
TD0 × G_1_	–7.46	0.762
TD2 × G_1_	30.95	0.206
TD0 × G_2_	–29.92	0.216
TD2 × G_2_	3.94	0.876
TD0 × G_3_	9.47	0.697
TD2 × G_3_	–14.42	0.562
TD0 × G_4_	10.18	0.673
TD2 × G_4_	–14.75	0.547

All coefficients, in milliseconds, of the LMM for the fixed factors in the model used to fit the gravitational timing error and the relative *P-value* values are shown (gravity condition G_0_, traveled distance TD1, visibility: occluded, and session order: occluded in the first block are the baseline). *P < 0.05.

**TABLE 9:** Effect of “catch trials” on hand motion duration.

	***Coeff***	***P*-value**
Intercept	25.50	0.088
TD0	2.40	0.909
TD2	–26.24	0.193
G_1_	–14.91	0.455
G_2_	–34.22	0.094
G_3_	–29.66	0.204
G_4_	–23.59	0.248
Visibility (V)	4.69	0.560
Session order (O)	2.57	0.732
TD0 × G_1_	–17.71	0.532
TD2 × G_1_	–7.26	0.797
TD0 × G_2_	26.99	0.333
TD2 × G_2_	41.09	0.157
TD0 × G_3_	4.08	0.884
TD2 × G_3_	58.39	0.042*
TD0 × G_4_	10.96	0.694
TD2 × G_4_	32.20	0.254

All coefficients in milliseconds of the LMM for the fixed factors in the model used to fit the timing error and the relative *P-value* values are shown (gravity condition G_0_, traveled distance TD1, visibility: occluded, and session order: occluded in the first block are the baseline). *P < 0.05.

The results showed that the movement temporization (e.g., both the TE and IT) did not depend on visibility while it depended on the gravity level. In particular, the movement was correctly timed only in G_0_. This is compatible with the hypothesis that participants timed the interception based on knowledge of the quantitative effects of Earth gravity during both the rolling and falling phases. In order to further test this hypothesis, we evaluated the TE and IT considering a hypothetical free-fall under natural gravity for all conditions.

#### Comparison With Free-Fall in Air Under Earth Gravity (After Natural or Unnatural Ball Rolling Motion on the Incline)

Consistent with the hypothesis that participants expected a free-fall in air at natural gravity irrespective of ball kinematics during the previous rolling phase, we found that the mean TE assuming a free-fall under natural gravity (GTE) was close to zero for all gravity conditions (Figure 10A). On average, GTE was -0.014 ± 0.016, -0.002 ± 0.021, -0.011 ± 0.012, -0.017 ± 0.017, and -0.014 ± 0.016 s (mean ± CI, *n* = 96, three traveled distances × two visual conditions × 16 subjects) for G_0_–G_4_. LMM (five gravity conditions, three traveled distances, twelve repetitions, two visual conditions, and two session order) showed that GTE did not depend significantly on gravity condition (all *P* > 0.083). Nor did GTE depend significantly on visibility, repetitions, and session order (Table 10).

**FIGURE 10:** Gravitational timing error and hand movement characteristics assuming a free-fall under natural gravity in air, instead of the actual kinematics. **A**–**D** in the same format as in Figure 8.

**TABLE 10:** Gravitational timing error.

	***Coeff***	***P*-value**
Intercept	–19.34	0.377
TD0	15.45	0.018*
TD2	–11.75	0.061
G_1_	14.42	0.083
G_2_	12.69	0.086
G_3_	2.39	0.659
G_4_	3.63	0.503
Visibility (V)	28.16	0.079
Session order (O)	6.03	0.704
Repetition	–1.83	0.201
TD0 × G_1_	0.11	0.998
TD2 × G_1_	–7.22	0.339
TD0 × G_2_	–10.47	0.162
TD2 × G_2_	–18.55	0.016*
TD0 × G_3_	–0.19	0.980
TD2 × G_3_	–13.22	0.081
TD0 × G_4_	–0.74	0.921
TD2 × G_4_	–8.90	0.240

All coefficients, in milliseconds, of the LMM for the fixed factors in the model used to fit the gravitational timing error and the relative *P-value* values are shown (gravity condition G_0_, traveled distance TD1, visibility: occluded, and session order: occluded in the first block are the baseline). *P < 0.05.

Figure 10C shows the top view of hand trajectories for all repetitions of one participant (same as in Figures 8C,D) for each gravity condition and traveled distance in the occluded session, considering a free-fall in air under natural gravity. The trajectories are plotted from the starting position to GIP. Consistent with the results relative to GTE, the *z*-coordinates of GIP were generally close to 0 (the *z*-coordinate of the frontal plane tangent to the ball surface facing the hitter), indicating a correct hand movement temporization for a target in free-fall under natural gravity. Figure 10B and Table 11 show that the time interval between the instant in which the hitter arrived in GIP and the maximum speed time did not depend on gravity conditions (with the exception of G_2_, *P* = 0.016). Figure 10D shows that the speed profiles for one subject (same as in Figures 8C,D) are well aligned on the arrival time of the hitter in GIP for all gravity conditions.

**TABLE 11:** Interval between the instant in which hitter arrived at instantaneous minimum distance from the ball surface considering ball gravitational free-fall (GIP), and the maximum speed time.

	***Coeff***	***P*-value**
Intercept	72.25	0.013*
TD0	–5.74	0.467
TD2	4.46	0.546
G_1_	–10.99	0.185
G_2_	–20.09	0.016*
G_3_	–6.61	0.288
G_4_	–0.67	0.913
Visibility (V)	–28.38	0.110
Session order (O)	–32.01	0.100
Repetition	2.09	0.077
TD0 × G_1_	12.59	0.137
TD2 × G_1_	–0.21	0.981
TD0 × G_2_	11.87	0.161
TD2 × G_2_	29.02	8.37−04***
TD0 × G_3_	6.74	0.425
TD2 × G_3_	17.89	0.037*
TD0 × G_4_	–1.43	0.866
TD2 × G_4_	6.29	0.463

All coefficients, in milliseconds, of the LMM for the fixed factors in the model used to fit the gravitational timing error and the relative *P-value* values are shown (gravity condition G_0_, traveled distance TD1, visibility: occluded, and session order: occluded in the first block are the baseline). *P < 0.05, ***P < 0.001.

## Discussion

We designed the experiments to test whether naturalness perception and interception timing are sensitive to the level of simulated gravity affecting the visual motion of a falling target. We specifically wanted to distinguish between three different hypotheses. (1) The internal model of Earth gravity accounts for a downward accelerated motion qualitatively, but does not discriminate between different gravity levels. (2) The internal model of gravity accounts for Earth gravitational kinematics quantitatively. (3) The prior model of ball motion can be updated by using online visual information of the rolling phase on the incline to predict the subsequent falling phase in air even for artificial gravity levels.

The results were generally compatible with the second hypothesis. Thus, perception rate of natural motion was significantly higher and less variable in G_0_ than in the other tested conditions, G_0_ being the only condition in which ball kinematics was congruent with Earth gravity during both the rolling phase and the free-falling phase. Moreover, on average, the timing of target interception was accurate in G_0_, late in G_2_ and G_4_ (when target acceleration prior to interception was higher than the expected value of Earth gravity), and early in G_1_ and G_3_ (when target acceleration was lower than the expected value).

Critically, neither the perceptual judgment of naturalness nor the interception timing depended significantly on whether or not the target was visible during free-fall. This latter result indicated that, even when occluded, free-fall under natural gravity was correctly extrapolated from the preceding, visible phase of rolling motion along the incline.

### Perceptual Judgments of Naturalness

The present results confirm and extend those of Ceccarelli et al. (2018). A visual scene including abundant static cues about the gravity reference and metric scale allows quantitative estimates of the effects of gravity on object motion, leading to perceptual judgments coherent with physics. This contrasts with the poor performance that is typically reported for perceptual estimates of naturalness of sloped motion in the absence of a structured visual context (Bozzi, 1959; Hecht, 1993; Rohrer, 2003). By the same token, discrimination of different gravity accelerations of parabolic motions presented against a blank background is low (Jörges et al., 2018). The present results, instead, are consistent with the suggestion put forth by Kaiser et al. (1985) that judgments of naturalness can be close to physical realism when the event to be judged is shown in motion. Smith et al. (2018) speculated that naturalness judgments require tracking and matching the precise position of an object over time, and therefore they might be well served by an analog simulation system (akin to an internal model of physics).

Here, naturalness perception depended on the motor performance, in addition to the gravity condition. Although motor performance by itself was related to the gravity condition, the absolute value of the TE of interception affected significantly the rate of naturalness judgments independently of the gravity condition: participants tended to judge more natural those target motions that they intercepted with smaller temporal errors. However, perceptual responses and motor responses were ranked in a slightly different order as a function of the gravity condition (compare Figures 5, 8A).

Motor performance could contribute to naturalness perception in different ways. First, since participants gave their judgments after performing the interception attempt, the mere action execution could have primed participants to be attuned to all available information about target kinematics, which, in turn, could have affected naturalness perception. Second, judgments of naturalness could be made with respect to the success of the interceptive action. In other words, the relative difficulty of interception and the corresponding error in motor timing could have prompted the participants to judge the event more or less natural.

Perceptual judgments cannot be disembodied from purposeful actions, implying that the manner with which a person interacts with a dynamic event provides a strong framework to judge critical features of the same event. In line of principle, motor actions might teach or shape perceptual skills. In particular, motor-perceptual interactions are to be expected when motor processes contribute to perception. For example, Ishimura and Shimojo (1994) reported a series of experiments where perceived motion was biased by concurrent hand movements. In another study, Wohlschläger (2000) showed that planned hand movements, which were performed only after the visual judgment, were sufficient to bias apparent motion perception. Likewise, Craighero et al. (1999) found that the mere preparation of reaching to grasp a bar in a certain orientation produced faster processing of stimuli congruent with bar orientation.

### Motor Control

The present results agree with those of Jörges and López-Moliner (2019) showing a quantitative relationship between the gravity level of a target moving along a parabolic path and the timing of button press responses. Notice that, also in the study of Jörges and López-Moliner (2019), the targets were presented against a background including different objects that allowed the metric calibration of space. In both studies, interception responses were timed correctly when target kinematics was congruent with Earth gravity, while the responses were early for gravity values lower than Earth gravity and late for gravity values higher than Earth gravity. Here, we found that the mean TE assuming a free-fall under natural gravity (GTE) was close to zero for all gravity conditions, further corroborating the hypothesis that participants expected a free-fall in air at natural gravity irrespective of ball kinematics during the previous rolling phase. Moreover, both the TEs and the parameters of hand movements did not depend significantly on target visibility during free-fall, demonstrating that ball kinematics during this phase was not simply extrapolated from the previous visible phase.

These findings are incompatible with the idea that the extrapolation of target motion is based only on the online visual information about target kinematics. The findings are in agreement with the previous studies that have already demonstrated the use of the internal model of gravity effects in interceptive actions in the presence of partial occlusion (Zago et al., 2010; Bosco et al., 2012; La Scaleia et al., 2014a, 2015). In particular, La Scaleia et al. (2015) performed an experiment reminiscent of the present one: participants were asked to hit a real ball that first rolled down an inclined plane tilted by 20° and then fell in air under Earth gravity and air drag along a quasi-parabolic trajectory, which was either visible or occluded. The interceptive performance was strikingly similar in the visual and occluded sessions, indicating that the internal model of gravity was used to extrapolate ball motion correctly even when this was occluded. Here, instead, we took advantage of the virtual reality setup to manipulate the ball acceleration for the motion on the inclined plane and for the motion in air independently. We found that online visual information about ball rolling motion was not used to update the model of the free-fall phase, which remained the model of a target falling under Earth gravity.

## Conclusion

The present results add to the growing evidence that, despite its poor sensitivity to generic visual accelerations, the brain is highly tuned to the specific kinematics associated with Earth gravity. Both perceptual and motor responses are guided by internal models of physics that allow the prediction of the forthcoming dynamics of events unfolding under gravity acceleration.

With regard to the issue of the design of virtual scenarios, we considered at the outset, one take-home message of the present study is that the rendering of animations should include realistic gravity effects along with contextual cues sufficient to calibrate the metrics of virtual space and motion. Instead, it does not seem necessary that visual information is complete and continuous, since human sensorimotor systems are capable of filling in huge gaps in the spatiotemporal unfolding of the stimuli (Bosco et al., 2015). Another take-home message of this study is that closing the sensorimotor loop, by asking the observer to interact with the target in the virtual scenario, enhances the perceptual sensitivity to physical realism. Therefore, vivid virtual environments should be as much interactive as possible, especially in view of designing physiologically inspired protocols for basic research and rehabilitation.

## Data Availability Statement

The datasets are available on request. The raw data supporting the conclusions of this article will be made available by the authors, without undue reservation, to any qualified researcher.

## Ethics Statement

The studies involving human participants were reviewed and approved by the Institutional Review Board of Santa Lucia Foundation. The patients/participants provided their written informed consent to participate in this study.

## Author Contributions

The work was performed at the Laboratory of Neuromotor Physiology, IRCCS Fondazione Santa Lucia. FC performed the experiments. BL, FC, and MZ analyzed the data. All authors conceived and designed research, and contributed to the interpretation of the data and drafting the work. All authors approved the final version of the manuscript, agreed to be accountable for all aspects of the work in ensuring that questions related to the accuracy or integrity of any part of the work are appropriately investigated and resolved, and that all persons designated as authors qualify for authorship, and all those who qualify for authorship are listed.

## Conflict of Interest

The authors declare that the research was conducted in the absence of any commercial or financial relationships that could be construed as a potential conflict of interest.

## References

[B1] BarraJ.SenotP.AuclairL. (2017). Internal model of gravity influences configural body processing. *Cognition* 158 208–214. 10.1016/j.cognition.2016.10.018 27842273

[B2] BohilC. J.AliceaB.BioccaF. A. (2011). Virtual reality in neuroscience research and therapy. *Nat. Rev. Neurosci.* 12 752–762. 10.1038/nrn3122 22048061

[B3] BootsmaR. J.Van WieringenP. C. (1990). Timing an attacking forehand drive in table tennis. *J. Exp. Psychol. Hum. Percept. Perform.* 16 21–29. 10.1037/0096-1523.16.1.21

[B4] BoscoG.Delle MonacheS.GravanoS.IndovinaI.La ScaleiaB.MaffeiV. (2015). Filling gaps in visual motion for target capture. *Front. Integr. Neurosci.* 9:13. 10.3389/fnint.2015.00013 25755637PMC4337337

[B5] BoscoG.Delle MonacheS.LacquanitiF. (2012). Catching what we can’t see: manual interception of occluded fly-ball trajectories. *PLoS One* 7:e49381. 10.1371/journal.pone.0049381 23166653PMC3498163

[B6] BozziP. (1959). Le condizioni del movimento “naturale” lungo i piani inclinati. *Riv. Psicol.* 53 337–352.

[B7] BozziP. (1961). Fenomenologia del movimento e dinamica pregalileiana. *Aut Aut* 64 1–24.

[B8] CalderoneJ. B.KaiserM. K. (1989). Visual acceleration detection: effect of sign and motion orientation. *Percept. Psychophys.* 45 391–394. 10.3758/bf03210711 2726400

[B9] Cano PorrasD.SiemonsmaP.InzelbergR.ZeiligG.PlotnikM. (2018). Advantages of virtual reality in the rehabilitation of balance and gait: systematic review. *Neurology* 90 1017–1025. 10.1212/WNL.0000000000005603 29720544

[B10] Cano PorrasD.ZeiligG.DonigerG. M.BahatY.InzelbergR.PlotnikM. (2019). Seeing gravity: gait adaptations to visual and physical inclines – A virtual reality study. *Front. Neurosci.* 13:1308 10.3389/fnins.2019.01308PMC699271132038123

[B11] CeccarelliF.La ScaleiaB.RussoM.CesquiB.GravanoS.MezzettiM. (2018). Rolling motion along an incline: visual sensitivity to the relation between acceleration and slope. *Front. Neurosci.* 12:406. 10.3389/fnins.2018.00406 29988401PMC6023988

[B12] ChambersC.FernandesH.KordingK. P. (2019). Policies or knowledge: priors differ between a perceptual and sensorimotor task. *J. Neurophysiol.* 121 2267–2275. 10.1152/jn.00035.2018 31017845PMC6620698

[B13] ChampagneA. B.KlopferL. E.AndersonJ. H. (1980). Factors influencing the learning of classical mechanics. *Am. J. Phys.* 48 1074–1079. 10.1119/1.12290

[B14] CraigheroL.FadigaL.RizzolattiG.UmiltàC. (1999). Action for perception: a motor-visual attentional effect. *J. Exp. Psychol. Hum. Percept. Perform.* 25 1673–1692. 10.1037/0096-1523.25.6.1673 10641315

[B15] DayB. L.LyonI. N. (2000). Voluntary modification of automatic arm movements evoked by motion of a visual target. *Exp. Brain Res.* 130 159–168. 10.1007/s002219900218 10672469

[B16] de RugyA.MarinovicW.WallisG. (2012). Neural prediction of complex accelerations for object interception. *J. Neurophysiol.* 107 766–771. 10.1152/jn.00854.2011 22090456

[B17] Delle MonacheS.LacquanitiF.BoscoG. (2019). Ocular tracking of occluded ballistic trajectories: effects of visual context and of target law of motion. *J. Vis.* 19:13. 10.1167/19.4.13 30952164

[B18] FranklinD. W.WolpertD. M. (2011). Computational mechanisms of sensorimotor control. *Neuron* 72 425–442. 10.1016/j.neuron.2011.10.006 22078503

[B19] GaveauJ.BerretB.AngelakiD. E.PapaxanthisC. (2016). Direction dependent arm kinematics reveal optimal integration of gravity cues. *eLife* 5:e16394. 10.7554/eLife.16394 27805566PMC5117856

[B20] GaveauJ.PaizisC.BerretB.PozzoT.PapaxanthisC. (2011). Sensorimotor adaptation of point-to-point arm movements after spaceflight: the role of internal representation of gravity force in trajectory planning. *J. Neurophysiol.* 106 620–629. 10.1152/jn.00081.2011 21562193

[B21] GoodaleM. A.MilnerA. D. (1992). Separate visual pathways for perception and action. *Trends Neurosci.* 15 20–25. 10.1016/0166-2236(92)90344-8 1374953

[B22] HechtH. (1993). Judging rolling wheels: dynamic and kinematic aspects of rotation – translation coupling. *Perception* 22 917–928. 10.1068/p220917 8190595

[B23] HubbardT. (ed.) (2018). *Spatial Biases in Perception and Cognition*. Cambridge: Cambridge University Press 10.1017/9781316651247

[B24] IndovinaI.MaffeiV.BoscoG.ZagoM.MacalusoE.LacquanitiF. (2005). Representation of visual gravitational motion in the human vestibular cortex. *Science* 308 416–419. 10.1126/science.1107961 15831760

[B25] IshimuraG.ShimojoS. (1994). “Voluntary action captures visual motion,” in *Proceedings of the Poster presented at the annual meeting of the Association for Research in Vision and Ophthalmology*, Sarasota, FL.

[B26] JeannerodM.ArbibM. A.RizzolattiG.SakataH. (1995). Grasping objects: the cortical mechanisms of visuomotor transformation. *Trends Neurosci.* 18 314–320. 10.1016/0166-2236(95)93921-j 7571012

[B27] JörgesB.HagenfeldL.López-MolinerJ. (2018). The use of visual cues in gravity judgements on parabolic motion. *Vis. Res.* 149:2018. 10.1016/j.visres.2018.06.002 29913247

[B28] JörgesB.López-MolinerJ. (2017). Gravity as a strong prior: implications for perception and action. *Front. Hum. Neurosci.* 11:203. 10.3389/fnhum.2017.00203 28503140PMC5408029

[B29] JörgesB.López-MolinerJ. (2019). Earth-gravity congruent motion facilitates ocular control for pursuit of parabolic trajectories. *Sci. Rep.* 9:14094. 10.1038/s41598-019-50512-6 31575901PMC6773720

[B30] KaiserM. K.ProffittD. R.AndersonK. (1985). Judgments of natural and anomalous trajectories in the presence and absence of motion. *J. Exp. Psychol. Learn. Mem. Cogn.* 11 795–803. 10.1037/0278-7393.11.1-4.795 2932526

[B31] KozhevnikovM.HegartyM. (2001). Impetus beliefs as default heuristics: dissociation between explicit and implicit knowledge about motion. *Psychonom. Bull. Rev.* 8 439–453. 10.3758/bf03196179 11700895

[B32] La ScaleiaB.LacquanitiF.ZagoM. (2014a). Neural extrapolation of motion for a ball rolling down an inclined plane. *PLoS One* 9:e99837. 10.1371/journal.pone.0099837 24940874PMC4062474

[B33] La ScaleiaB.ZagoM.LacquanitiF. (2015). Hand interception of occluded motion in humans: a test of model-based vs. on-line control. *J. Neurophysiol.* 114 1577–1592. 10.1152/jn.00475.2015 26133803PMC4563024

[B34] La ScaleiaB.ZagoM.MoscatelliA.LacquanitiF.VivianiP. (2014b). Implied dynamics biases the visual perception of velocity. *PLoS One* 9:e93020. 10.1371/journal.pone.0093020 24667578PMC3965519

[B35] LacquanitiF.BoscoG.IndovinaI.La ScaleiaB.MaffeiV.MoscatelliA. (2013). Visual gravitational motion and the vestibular system in humans. *Front. Integr. Neurosci.* 7:101. 10.3389/fnint.2013.00101 24421761PMC3872780

[B36] LacquanitiF.CarrozzoM.BorgheseN. A. (1993). “The role of vision in tuning anticipatory motor responses of the limbs,” in *Multisensory Control of Movement*, ed. BerthozA. (Oxford: Oxford University Press), 379–393. 10.1093/acprof:oso/9780198547853.003.0190

[B37] LacquanitiF.MaioliC. (1989a). Adaptation to suppression of visual information during catching. *J. Neurosci.* 9 149–159. 10.1523/jneurosci.09-01-00149.1989 2913201PMC6570000

[B38] LacquanitiF.MaioliC. (1989b). The role of preparation in tuning anticipatory and reflex responses during catching. *J. Neurosci.* 9 134–148. 10.1523/jneurosci.09-01-00134.1989 2913200PMC6570012

[B39] LeeD. N.YoungD. S.ReddishP. E.LoughS.ClaytonT. M. (1983). Visual timing in hitting an accelerating ball. *Q. J. Exp. Psychol. A* 35 333–346. 10.1080/14640748308402138 6571315

[B40] MaffeiV.IndovinaI.MacalusoE.IvanenkoY. P.OrbanG.LacquanitiF. (2015). Visual gravity cues in the interpretation of biological movements: neural correlates in humans. *Neuroimage* 104 221–230. 10.1016/j.neuroimage.2014.10.006 25315789

[B41] MarinovicW.PlooyA. M.TresilianJ. R. (2009). Preparation and inhibition of interceptive actions. *Exp. Brain Res.* 197 311–319. 10.1007/s00221-009-1916-0 19565223

[B42] McIntyreJ.ZagoM.BerthozA.LacquanitiF. (2001). Does the brain model Newton’s laws? *Nat. Neurosci.* 4 693–694. 10.1038/89477 11426224

[B43] McLeodP. (1987). Visual reaction time and high-speed ball games. *Perception* 16 49–59. 10.1068/p160049 3671040

[B44] MichaelsC. F.ZeinstraE. B.OudejansR. R. (2001). Information and action in punching a falling ball. *Q. J. Exp. Psychol. A* 54 69–93. 10.1080/02724980042000039 11216322

[B45] MillerW. L.MaffeiV.BoscoG.IosaM.ZagoM.MacalusoE. (2008). Vestibular Nuclei and Cerebellum Put Visual Gravitational Motion in Context. *J. Neurophysiol.* 99 1969–1982. 10.1152/jn.00889.2007 18057110

[B46] MischiatiM.LinH.-T.HeroldP.ImlerE.OlbergR.LeonardoA. (2015). Internal models direct dragonfly interception steering. *Nature* 517 333–338. 10.1038/nature14045 25487153

[B47] MiwaT.HisakataR.KanekoH. (2019). Effects of the gravity direction in the environment and the visual polarity and body direction on the perception of object motion. *Vis. Res.* 164 12–23. 10.1016/j.visres.2019.08.005 31542657

[B48] MoscatelliA.La ScaleiaB.ZagoM.LacquanitiF. (2019). Motion direction, luminance contrast, and speed perception: an unexpected meeting. *J. Vis.* 19:16. 10.1167/19.6.16 31206138

[B49] MoscatelliA.LacquanitiF. (2011). The weight of time: gravitational force enhances discrimination of visual motion duration. *J. Vis.* 11:5. 10.1167/11.4.5 21478379

[B50] MoscatelliA.MezzettiM.LacquanitiF. (2012). Modeling psychophysical data at the population-level: the generalized linear mixed model. *J. Vis.* 12:26. 10.1167/12.11.26 23104819

[B51] MrotekL. A.SoechtingJ. F. (2007). Predicting curvilinear target motion through an occlusion. *Exp. Brain Res.* 178 99–114. 10.1007/s00221-006-0717-y 17053910

[B52] PortN. L.LeeD.DassonvilleP.GeorgopoulosA. P. (1997). Manual interception of moving targets. I. Performance and movement initiation. *Exp. Brain Res.* 116 406–420. 10.1007/pl00005769 9372290

[B53] R Development Core Team (2011). *R: A Language and Environment for Statistical Computing*. Vienna: R Foundation for Statistical Computing.

[B54] RebenitschL.OwenC. (2016). Review on cybersickness in applications and visual displays. *Virtual Real.* 20 101–125. 10.1007/s10055-016-0285-9

[B55] RohrerD. (2003). The natural appearance of unnatural incline speed. *Mem. Cogn.* 31 816–826. 10.3758/BF03196119 12956245

[B56] RussoM.CesquiB.La ScaleiaB.CeccarelliF.MaselliA.MoscatelliA. (2017). Intercepting virtual balls approaching under different gravity conditions: evidence for spatial prediction. *J. Neurophysiol.* 118 2421–2434. 10.1152/jn.00025.2017 28768737PMC5646193

[B57] Sanchez-VivesM. V.SlaterM. (2005). From presence to consciousness through virtual reality. *Nat. Rev. Neurosci.* 6 332–339. 10.1038/nrn1651 15803164

[B58] SenotP.ZagoM.LacquanitiF.McIntyreJ. (2005). Anticipating the effects of gravity when intercepting moving objects: differentiating up and down based on nonvisual cues. *J. Neurophysiol.* 94 4471–4480. 10.1152/jn.00527.2005 16120661

[B59] SenotP.ZagoM.Le Séac’hA.ZaouiM.BerthozA.LacquanitiF. (2012). When up is down in 0g: how gravity sensing affects the timing of interceptive actions. *J. Neurosci.* 32 1969–1973. 10.1523/JNEUROSCI.3886-11.2012 22323710PMC6621712

[B60] ShanonB. (1976). Aristotelianism, Newtonianism and the physics of the layman. *Perception* 5 241–243. 10.1068/p050241 951174

[B61] SmithK. A.BattagliaP. W.VulE. (2018). Different physical intuitions exist between tasks, not domains. *Comput. Brain Behav.* 1 101–118. 10.1007/s42113-018-0007-3

[B62] SveistrupH. (2004). Motor rehabilitation using virtual reality. *J. Neuroeng. Rehabil.* 1:10. 1567994510.1186/1743-0003-1-10PMC546406

[B63] TecchiaF.CarrozzinoM.BacinelliS.RossiF.VercelliD.MarinoG. (2010). A flexible framework for wide-spectrum VR development. *Presence* 19 302–312. 10.1162/pres_a_00002

[B64] TramperJ. J.LamontA.FlandersM.GielenS. (2013). Gaze is driven by an internal goal trajectory in a visuomotor task. *Eur. J. Neurosci.* 37 1112–1119. 10.1111/ejn.12107 23279153PMC3618614

[B65] TresilianJ. R. (1995). Perceptual and cognitive processes in time-to-contact estimation: analysis of prediction-motion and relative judgment tasks. *Percept. Psychophys.* 57 231–245. 10.3758/bf03206510 7885822

[B66] TresilianJ. R. (1997). Revised tau hypothesis: a consideration of Wann’s (1996) analyses. *J. Exp. Psychol. Hum. Percept. Perform.* 23 1272–1281. 10.1037/0096-1523.23.4.1272

[B67] TrojeN. F.ChangD. H. F. (2013). “Shape-independent processing of biological motion,” in *People Watching: Social, Perceptual, and Neurophysiological Studies of Body Perception*, eds JohnsK. L.ShiffrarM. (Oxford: Oxford University Press), 82–100. 10.1093/acprof:oso/9780195393705.003.0006

[B68] van SoestA. J. K.CasiusL. J. R.de KokW.KrijgerM.MeederM.BeekP. J. (2010). Are fast interceptive actions continuously guided by vision? Revisiting Bootsma and van Wieringen (1990). *J. Exp. Psychol. Hum. Percept. Perform.* 36 1040–1055. 10.1037/a0016890 20695717

[B69] VicarioG. B.BressanP. (1990). Wheels: a new illusion in the perception of rolling objects. *Perception* 19 57–61. 10.1068/p190057 2336336

[B70] VicovaroM. (2014). Intuitive physics of free fall: an information integration approach to the mass-speed belief. *Psicol. Int. J. Methodol. Exp. Psychol.* 35 463–477.

[B71] VicovaroM.NoventaS.BattagliniL. (2019). Intuitive physics of gravitational motion as shown by perceptual judgment and prediction-motion tasks. *Acta Psychol.* 194 51–62. 10.1016/j.actpsy.2019.02.001 30743090

[B72] VishtonP. M.ReardonK. M.StevensJ. A. (2010). Timing of anticipatory muscle tensing control: responses before and after expected impact. *Exp. Brain Res.* 202 661–667. 10.1007/s00221-010-2172-z 20135099

[B73] WerkhovenP.SnippeH. P.ToetA. (1992). Visual processing of optic acceleration. *Vis. Res.* 32 2313–2329. 10.1016/0042-6989(92)90095-z 1288008

[B74] WohlschlägerA. (2000). Visual motion priming by invisible actions. *Vis. Res.* 40 925–930. 10.1016/s0042-6989(99)00239-4 10720663

[B75] ZagoM.BoscoG.MaffeiV.IosaM.IvanenkoY. P.LacquanitiF. (2004). Internal models of target motion: expected dynamics overrides measured kinematics in timing manual interceptions. *J. Neurophysiol.* 91 1620–1634. 10.1152/jn.00862.2003 14627663

[B76] ZagoM.IosaM.MaffeiV.LacquanitiF. (2010). Extrapolation of vertical target motion through a brief visual occlusion. *Exp. Brain Res.* 201 365–384. 10.1007/s00221-009-2041-9 19882150

[B77] ZagoM.La ScaleiaB.MillerW. L.LacquanitiF. (2011). Coherence of structural visual cues and pictorial gravity paves the way for interceptive actions. *J. Vis.* 11 13–13. 10.1167/11.10.13 21933933

[B78] ZagoM.LacquanitiF. (2005). Cognitive, perceptual and action-oriented representations of falling objects. *Neuropsychologia* 43 178–188. 10.1016/j.neuropsychologia.2004.11.005 15707903

[B79] ZagoM.McIntyreJ.SenotP.LacquanitiF. (2009). Visuo-motor coordination and internal models for object interception. *Exp. Brain Res.* 192 571–604. 10.1007/s00221-008-1691-3 19139857

